RETRACTED

# Mapping C-Terminal Transactivation Domains of the Nuclear HER Family Receptor Tyrosine Kinase HER3

**DOI:** 10.1371/journal.pone.0071518

**Published:** 2013-08-08

**Authors:** Toni M. Brand, Mari Iida, Neha Luthar, Matthew J. Wleklinski, Megan M. Starr, Deric L. Wheeler

**Affiliations:** Department of Human Oncology, University of Wisconsin School of Medicine and Public Health, Madison, Wisconsin, United States of America; University of Geneva, Switzerland

## Abstract

Nuclear localized HER family receptor tyrosine kinases (RTKs) have been observed in primary tumor specimens and cancer cell lines for nearly two decades. Inside the nucleus, HER family members (EGFR, HER2, and HER3) have been shown to function as co-transcriptional activators for various cancer-promoting genes. However, the regions of each receptor that confer transcriptional potential remain poorly defined. The current study aimed to map the putative transactivation domains (TADs) of the HER3 receptor. To accomplish this goal, various intracellular regions of HER3 were fused to the DNA binding domain of the yeast transcription factor Gal4 (Gal4DBD) and tested for their ability to transactivate Gal4 UAS-luciferase. Results from these analyses demonstrated that the C-terminal domain of HER3 (CTD, amino acids distal to the tyrosine kinase domain) contained potent transactivation potential. Next, nine HER3-CTD truncation mutants were constructed to map minimal regions of transactivation potential using the Gal4 UAS-luciferase based system. These analyses identified a bipartite region of 34 (B_1_) and 27 (B_2_) amino acids in length that conferred the majority of HER3’s transactivation potential. Next, we identified full-length nuclear HER3 association and regulation of a 122 bp region of the cyclin D1 promoter. To understand how the B_1_ and B_2_ regions influenced the transcriptional functions of nuclear HER3, we performed cyclin D1 promoter-luciferase assays in which HER3 deleted of the B_1_ and B_2_ regions was severely hindered in regulating this promoter. Further, the overexpression of HER3 enhanced cyclin D1 mRNA expression, while HER3 deleted of its identified TADs was hindered at doing so. Thus, the ability for HER3 to function as a transcriptional co-activator may be dependent on specific C-terminal TADs.

## Introduction

The ErbB/HER family of receptor tyrosine kinases (RTKs) consists of four family members: the epidermal growth factor receptor (EGFR/ErbB1), HER2 (ErbB2/Neu), HER3 (ErbB3), and HER4 (ErbB4). This family of RTKs has been highly implicated in the formation and progression of various cancers via aberrant overexpression, kinase activation, and mutation [1], [2]. Classically, HER family members function from the cell surface, where binding to cognate ligands can induce receptor homo- or hetero-dimerization with other HER family receptors [3]. The HER2 receptor does not bind to any known ligands, however, its dimerization arm is innately positioned in an open conformation. This process leads to the activation of each receptors’ tyrosine kinase and the subsequent phosphorylation of tyrosine residues located on their C-terminal tails. Phosphorylated tyrosine residues recruit various intracellular adaptor and effector molecules that result in the propagation of growth promoting signal transduction cascades [1], [2]. Membrane-bound HER receptors activate numerous tumor promoting signaling cascades via this mechanism, including the PI3K/AKT, Ras/Raf/Mek/Erk, PLCγ/PKC, and signal transducer and activator of transcription (STAT) pathways [1], [2].

RETRACTED

While the classical membrane-bound functions of HER family RTKs have been extensively studied, accumulating data suggest that these receptors can be found in the cell’s nucleus where they can function as co-transcriptional activators [4], [5]. To date, EGFR, HER2, and a nuclear variant of HER3 have been shown to function as co-transcriptional activators for cyclin D1 [6]–[8]. Clinically, nuclear EGFR has been correlated with poor overall survival in breast [9], [10], ovarian [11], oropharyngeal [9], [12], and gallbladder [13] cancers. Nuclear EGFR has also been shown to play a role in resistance to numerous cancer therapies, including radiation [14]–[18], cisplatin [17]–[19], and the anti-EGFR therapies cetuximab [20] and gefitinib [21]. Collectively, these pivotal studies suggest that nuclear HER family receptors may enhance the tumorigenic phenotype of cancer cells, and therefore their nuclear roles must be further elucidated.

The HER3 receptor has recently come to the forefront as playing a key role in HER family driven cancers [22], [23]. HER3 is a unique HER family member in that it has diminished tyrosine kinase activity due to the lack of specific amino acids within its kinase domain [24], [25]. However, HER3 plays a crucial role as an allosteric activator of other HER family members in addition to functioning as a signaling substrate through the direct recruitment and activation of PI3K [26], [27]. With the discovery of the various functions of nuclear EGFR and HER2, recent interest has prompted the investigation of nuclear HER3. HER3 was first identified to be nuclear localized in normal and malignant mammary epithelial cells in 2002 [28]. HER3 was also shown to be prominently nuclear localized in malignant prostate cancer tissues, where it was correlated with risk of disease progression [29]. Most recently, two nuclear C-terminal splice variants of HER3 were identified and shown to function as co-transcriptional activators [8], [30]. Thus, the functions of nuclear HER3 are just beginning to unfold.

RETRACTED

In the current study we focused on identifying the amino acid regions on the C-terminal tail of HER3 that function as transactivation domains (TADs). First, numerous cancer cell lines were characterized for the expression of HER3, which was prominently nuclear localized in its full-length form. Next, various HER3 intracellular cytoplasmic domain (ICD) regions fused to the Gal4 DNA binding domain (Gal4DBD) were analyzed, and the C-terminal domain (CTD, amino acids distal to the tyrosine kinase domain) of HER3 was shown to activate the Gal4 upstream activation sequence (UAS) fused to luciferase. To identify specific C-terminal TADs, we created nine HER3-CTD truncation mutants and identified a bipartite region of 34 and 27 amino acids in length (denoted as B_1_ and B_2_) that contained the majority of HER3’s transactivation potential. To determine if the identified B_1_ and B_2_ TADs could augment nuclear HER3’s transcriptional function in cells, we first identified that full-length nuclear HER3 could associate and activate a 122 bp region of the cyclin D1 promoter when overexpressed. Importantly, the overexpression of HER3 lacking the B_1_ and B_2_ regions was severely hindered both in activating the 122 bp region of the cyclin D1 promoter and in enhancing transcription from the endogenous cyclin D1 gene. Collectively, these data suggest that this bipartite region of HER3 functions as a prominent TAD to mediate HER3’s nuclear functions.

## Materials and Methods

### Cell Lines

The human breast cancer cell line MCF-7, human colorectal cancer (CRC) cell lines LoVo, CaCO2, and CHOK1 cells were purchased from ATCC (Manassas, VA, USA). The human NSCLC line NCI-H226^R^ was developed as a cetuximab resistant cell line previously described [31], [32]. The human breast cancer cell lines SKBr3, BT474, HCC1954, and BT549 were kindly supplied by Dr. J. Boerner (Wayne State University School of Medicine, Karmanos Cancer Institute, MI, USA) [33], the human NSCLC cell line H522 was kindly supplied by Dr. R. Salgia (The University of Chicago Medical Center, IL, USA) [34], and human HNSCC cell lines SCC-1 and SCC-6 were kindly supplied by Dr. T. Carey (University of Michigan, MI, USA) [35]. All cell lines were maintained in their respective media with 10% fetal bovine serum and 1% penicillin and streptomycin; SKBr3, BT549, SCC-1, and SCC-6 were maintained in Dulbecco’s modified Eagle’s medium (Mediatech Inc., Manassas, VA, USA); BT474, HCC1954, and H226^R^ were maintained in RPMI 1640 (Mediatech Inc.); CaCO2 was maintained in minimum essential medium eagle (Mediatech Inc.); LoVo and CHOK1 cells were maintained in F12K medium (Mediatech Inc.); MCF-7 cells were maintained in DMEM/F12K medium (Mediatech Inc.).

RETRACTED

### Antibodies and Compounds

All antibodies were obtained from the following sources: HER3-C- TERM (SC-285), HER3-N-TERM (SC-292557), Histone H3 (SC-28654), EGFR (SC-03), HER2 (SC-284), Gal4DBD (SC-510), HRP-conjugated goat-anti-rabbit IgG, and HRP-conjugated goat-anti mouse IgG were purchased from Santa Cruz Biotechnology Inc. (Santa Cruz, CA, USA). EGFR (1902-1, EP38Y) was purchased from Epitomics/Abcam (Cambridge, MA, USA). pHER3-Y1222 (#4784), pHER3-Y1289 (#4791), and GAPDH (#2118) were purchased from Cell Signaling Technology (Beverly, MA, USA). α-tubulin was purchased from Calbiochem (San Diego, CA, USA). Neuregulin-1 (NRG) was purchased from R&D Systems (Minneapolis, MN, USA).

### Cellular Fractionation and Immunoblotting Analysis

Cellular fractionation was performed as previously described [6], [36]. Cells were plated in either 10 cm or 15 cm dishes. At ∼80–90% confluency, cells were scraped in PBS and swelled in cytoplasmic lysis buffer (20 mM HEPES, pH 7.0, 10 mM KCl, 2 mM MgCl_2_, 0.5% NP40, 1 mM Na_3_VO_4_, 1 mM PMSF, 1 mM β-glycerophosphate (BGP), 10 ug/ml of leupeptin and aprotinin) for 15 min on ice. Cells were then homogenized by 30–40 strokes in a tightly fitting Dounce homogenizer and checked under microscope for intact nuclei. The homogenate was centrifuged at 1,500 g for 5 min at 4°C to sediment the nuclei. The nuclear pellet was washed 5 times in cytoplasmic lysis buffer to ensure complete removal of cytosolic membranes. After washes, the nuclear pellet was lysed in the same buffer with the addition of 0.5 M NaCl. Nuclear pellets were sonicated for 10 sec, and vortexed for 30 sec 3 times. The extracted nuclear lysate was centrifuged at 15,000 g for 10 min at 4°C, and the supernatants were collected as nuclear lysate. Whole cell protein lysate was obtained through lysis with RIPA buffer (50 mM HEPES, pH 7.4, 150 mM NaCl,.1% Tween-20, 10% glycerol, 2.5 mM EGTA, 1 mM EDTA, 1 mM DTT, 1 mM Na_3_VO_4,_ 1 mM PMSF, 1 mM BGP, and 10 ug/ml of leupeptin and aprotinin). Samples were sonicated for 10 sec, and then centrifuged at 15,000 g for 10 min at 4°C. All protein lysates were quantified by Bradford assay (Bio-Rad Laboratories, Hercules, CA, USA). Equal amounts of protein (∼20 ug) were fractionated by SDA-PAGE, transferred to a PVDF membrane (Millipore, Billerica, MA, USA), and analyzed by incubation with the appropriate primary antibody overnight at 4°C. Membranes were then subjected to incubation with HRP-conjugated secondary antibodies for 1 hr at room temperature. ECL chemiluminescence detection system was used to visual proteins with either of the following reagents: ECL Western Blotting Substrate (Promega Cooperation, Madison, WI, USA) or SuperSignal West Dura Extended Duration Chemiluminescent Substrate (Thermo Fisher Scientific, Walham, MA, USA).

RETRACTED

### Immunoprecipitation of HER3

Cells were lysed with NP-40 lysis buffer (50 mM HEPES, pH 7.4, 150 mM NaCl, 1% NP-40, 0.5% Deoxycholic acid, 10% glycerol, 2.5 mM EGTA, 1 mM EDTA, 1 mM DTT, 1 mM PMSF, 1 mM BGP, 1 mM Na_3_VO_4,_ and 10 ug/ml of leupeptin and aprotinin). Lysates were sheered via syringe 3 times, and then centrifuged at 15,000 g for 10 min at 4°C. 250 ug of protein was incubated overnight at 4°C with 2 ug of primary C-TERM or N-TERM HER3 antibody. Normal human IgG (Sigma, St. Louis, MO) was used as a negative control. Next day, 25 ul of protein A/G agarose beads (Santa Cruz Biotechnology) were added for 3 hr at 4°C. The immunoprecipitates were pelleted by centrifugation and washed 5 times with NP-40 lysis buffer. The captured immunocomplexes were eluted by boiling in 2×SDS sample buffer for 5 min and subjected to immunoblot analysis as described above.

### Immunofluorescent Staining of HER3

Approximately 3×10^3^ cells/well were seeded on a four-well glass chamber slide (Millipore). 24 hr later, cells were washed briefly with PBS, and fixed with 4% methanol-free formaldehyde for 15 min at room temperature. Cells were rinsed with PBS again, and permeabilized with PBS containing 0.2% TritonX-100 for 15 min. Cells were blocked in 5% normal goal serum diluted in PBS containing 0.3% Triton X-100 for 1 hr at room temperature, and primary C-TERM or N-TERM HER3 antibody was incubated overnight at 4°C. The next day, cells were rinsed with PBS 3 times, and incubated with Alexa Fluor-546 rabbit secondary antibody for 30 min at room temperature (Life Technologies, Carlsbad, CA, USA). Cells were rinsed with PBS again and mounted with ProLong gold with DAPI antifade mounting solution (Life Technologies). Fluorescence microscopy and photography were performed using a Nikon 80 i upright confocal microscope.

### Plasmid Construction and Transfection

Wild-type human HER3-pSPORT6 vector was kindly provided to us by Dr. P. Bertics (University of Wisconsin-Madison, WI, USA). HER3 was subsequently amplified via polymerase chain reaction and subcloned into KpnI/NotI restriction sites of the pcDNA6/V5-HisA vector (Life Technologies). PCDNA3.0-EGFRWT was kindly supplied by Dr. J. Boerner (Wayne State University School of Medicine, Karmanos Cancer Institute, MI, USA). EGFR-ICD and CTD, and HER3-ICD, JKD, and CTD were cloned into the pM-Gal4DBD expression vector using the SmaI/XbaI restriction sites (Clontech, Mountain View, CA, USA). Gal4DBD-EGFR, Gal4DBD-HER3, pcDNA6-HER3, pcDNA6-HER3ΔB_1_B_2_, pcDNA6-HER3WT-ICD, and pcDNA6-HER3ΔB_1_B_2_-ICD constructs were generated using the Phusion Site-Directed Mutagenesis Kit (Finnzymes, Keilaranta, Finland). pSPORT6-HER3-Y1222F/Y1289F construct was created via QuikChange II XL Site-Directed Mutagenesis Kit (Stratagene, La Jolla, CA, USA) following the manufacturer’s instructions. All mutations were verified for correct orientation and integrity via sequencing. The pGL4.35[luc2P/9XGal4UAS/Hygro], pGL3-Basic-Luciferase, and pRL-Tk-*Renilla* vectors were purchased from Promega. The 122 bp region of the cyclin D1 promoter (−33− +89) was subcloned into the pGL3-Basic promoterless vector using the KpnI/HindIII restriction sites. The sequences for this primer set are the following: CyD1 FWD 5′-CGGGGTACCCCGGGCTT GATCTTTGCT-3′, CyD1 REV 5′-CCCAAGCTTGACTCTGCTGCTCGCTGCTA-3′.

RETRACTED

All plasmid transfections were performed using Lipofectamine LTX and Opti-MEM I (Life Technologies) according to the manufacturer’s instructions. Cells were analyzed 24–72 hr post transfection for protein, luciferase activity, and mRNA. For siRNAs, cells were transfected with siHER3 (ON-TARGETplus SMARTpool HER3, L-003127 Dharmacon, Lafayette, CO, USA) or siNon-targeting (NT) (ON-TARGETplus Non-targeting Pool, D-001810, Dharmacon) using Lipofectamine RNAiMAX (Life Technologies) according to the manufacturer’s instructions. Vehicle (V) treated cells were treated with RNAiMAX only. For luciferase studies post siRNA, cells were transfected 24 hr later with cyclin D1-luciferase and *Renilla* plasmids, and analyzed for luciferase activity 48 hr later. For protein analysis, cells were lysed 72 hr post transfection and analyzed via western blot for HER3 knockdown.

### Luciferase Assay

Cells were plated in 6-well plates at approximate 70% confluence. For the Gal4 UAS-luciferase assay, cells were transiently transfected with 100 ng plasmid DNA, 1 ug of pGL4.35 Gal4 UAS-luciferase vector (Promega), and 100 ng of pRL-Tk-*Renilla* vector (Promega). For the cyclin D1 promoter luciferase assay, 2 ug of HER3 expression vectors, 1 ug of the 122 bp cyclin D1 promoter-pGL3 luciferase construct, and 10–100 ng of pRL-Tk-*Renilla* vector (Promega) were used. 48 hr post transfection, cells were collected for analysis via the Dual-Luciferase Reporter Assay System (Promega) according to the manufacturer’s protocol. Both *Firefly* and *Renilla* luciferase reporters were detected in a 96 well format using a Synergy 2 Multi-Mode Microplate Reader (BioTek, Winooski, VT, USA). Transfection efficiencies were normalized against DNA content, protein content, and the expression of *Renilla* Luciferase.

RETRACTED

### Chromatin Immunoprecipitation (ChIP)

Cells were plated in 15 cm plates at ∼80% confluency in quadruplicate. Each plate was fixed with formaldehyde at a final concentration of 1% for 15 min at room temperature. Fixation was terminated via 1.25 M glycine for 5 min, and cells were subsequently scraped in ice-cold PBS with 1 mM of PMSF. The cells were pelleted by centrifugation at 1500 rpm for 5 min at 4°C and then lysed in cell lysis buffer (5 mM HEPES, pH 8.0, 85 mM KCl, 0.5% NP-40 and 10 mM sodium pyrophosphate). 10 min later cells were further homogenized via Dounce homogenizer (30 strokes), and centrifuged for 1500 g for 5 min at 4°C. The supernatant was removed and nuclei pellets were lysed in nuclei lysis buffer (Tris-HCl 50 mM, pH 8.1, 10 mM EDTA, 1% SDS and 10 mM sodium pyrophosphate). The lysate was sonicated on ice for varied time points to achieve ∼500 bp fragments of DNA (sonication was optimized via running sheared DNA on 1% agarose gels). The supernatant was pre-cleared with protein A/G agarose beads (Santa Cruz Biotechnology) in dilution buffer (16.7 mM Tris-HCl, pH 8.1, 1.2 mM EDTA, 167 mM NaCl, 1.1% Triton X-100, 0.01% SDS and 10 mM sodium pyrophosphate) for 1 hr at 4°C. The pre-cleared lysates were immunoprecipated by incubating with protein A/G beads containing 5 ug of the N-TERM anti-HER3 antibody or human IgG (Sigma) rotating overnight at 4°C. The next day immunocomplexes were centrifuged at 1500 rpm for 5 min, and the beads were washed via light vortex for 15 min time intervals with the following wash buffers: wash buffer I (25 mM Tris-HCl, pH 8.0, 2 mM EDTA, 150 mM NaCl, 1% Triton X-100, 0.1% SDS and 10 mM sodium pyrophosphate), wash buffer II (25 mM Tris-HCl, pH 8.0, 2 mM EDTA, 500 mM NaCl, 1% Triton X-100, 0.1% SDS and 10 mM sodium pyrophosphate), wash buffer III (10 mM Tris-HCl, pH 8.0, 1 mM EDTA, 250 mM LiCl, 1% NP-40, 1% deoxycholic acid and 10 mM sodium pyrophosphate), and TE buffer (10 mM Tris-HCl, pH8.0, 1 mM EDTA, 10 mM sodium pyrophosphate). The bound DNA was eluted twice with elution buffer (10 mM NaHCO_3_ and 1% SDS). 5 mM NaCl was then added to the pooled DNA and incubated at 68°C overnight. The DNA was recovered and purified using a DNA purification kit (Qiagen, Valencia, CA, USA). The purified chromatin-immunoprecipitated DNA was used as template for qPCR with primers flanking the 122 bp region (−33− +89) of the cyclin D1 promoter: Cyclin D1 FWD 5′-CCGGGCTTGATCTTTGCT-3′, Cyclin D1 REV 5′-GACTCTGCTGCTCGCTGCTA-3′. The qPCR program was: 95°C for 3 min, followed by 40 cycles of 95°C for 15 sec and 55.5°C for 30 sec. The qPCR was performed using the CFX96 Real-Time PCR Detection System (Bio-Rad Laboratories).

RETRACTED

### DNA Affinity Pull Down Assay (DAPA)

DAPA was performed as previously described [37]. The nucleotide sequences of the 5′ biotinylated oligonucleotides corresponding to the 122 bp cyclin D1 promoter (−33− +89) are the following: Sense 5′- CCGGGCTTGATCTTTGCTTAACAACAGTAACGTCACACGGACTACAGGGGAGTTTTGTTGAAGTTGCAAAGTCCTGGAGCCTCCAGAGGGCTGTCGGCGCAGTAGCAGCGAGCAGCAGAGTC-3′, and Antisense 5′-GACTCTGCTGCTCGCTGCTACTGCGCCGACAGCCCTCTGGAGGCTCCAGGACTTTGCAACTTCAACAAAACTCCCCTGTAGTCCGTGTGACGTTACTGTTGTTAAGCAAAGATCAAGCCCGG-3′. The probes were purchased from Integrated DNA Technologies (Coralville, IA, USA). Following annealing of Sense and Anti-sense oligonucleotdies for 1 hr at 95°C, 4 ug of annealed biotinylated probe was incubated with 500 ug of nuclear cell lysate, and 40 ul of streptavidin-agarose bead suspension (Sigma) in PBS diluted with 1 mM Na_3_VO_4_, 1 mM PMSF, 1 mM BGP, 10 ug/ml of leupeptin and aprotinin for 2–3 hr rocking at room temperature. The streptavidin-agarose beads were pelleted by centrifugation and washed 5 times with PBS. The captured probe binding proteins were eluted from the streptavidin-agarose beads by boiling in 2×SDS sample buffer for 5 min and subjected to immunoblot analysis for HER3 binding.

### cDNA Synthesis and Quantitative PCR

Total RNA from cells was prepared using an RNeasy Mini kit (Qiagen, Inc., Valencia, CA). cDNA from total RNA of cells was synthesized using qScript cDNA SuperMix (Quanta BioSciences, Inc., Gaithersburg, MD, USA) according to manufacturer’s protocol. qPCR analysis was performed using a Bio-Rad CFX96 Real-Time PCR Detection System (Bio-Rad Laboratories). The primer sets used for this analysis were purchased from Life Technologies TaqMan® Gene Expression Assay: Cyclin D1 (Hs00765553_m1) and β-actin (Hs99999903_m1). For amplification cDNA was combined with primers and TaqMan universal PCR Master Mix (Life Technologies) according to the manufacturer’s instructions. All reactions were performed in triplicate. To determine the normalized value, 2^−ΔΔCt^ values were compared between cyclin D1 and endogenous control (β-actin) samples, where the change in crossing threshold (ΔCt) = Ct_Cyclin D1_-Ct_β-actin_ and ΔΔCt = ΔCt_(HER3WT or HER3ΔB1ΔB2)_-ΔCt_(Vector)_.

### Statistical Analysis

Student t-tests were used to evaluate the significance of changes in all reporter and expression assays as compared to vector only or non-targeting controls. Statistical analysis comparing antibody pull downs in all ChIP assays were also evaluated via Student t-test. Differences were considered statistically significant if *P*≤0.05.

RETRACTED

## Results

### The HER3 Receptor is Localized to the Nucleus in its Full-length Form

The overexpression of the HER3 receptor has been observed in cancers of the breast [38], non-small cell lung (NSCLC) [39], head and neck (HNSCC) [40], and colon (CRC) [41]. Therefore various cell lines from each cancer type were probed for HER3 expression, including the breast cancer cell lines SKBr3, MCF-7, BT474, HCC1954, and BT549, NSCLC cell lines H522 and H226^R^ (a cell line previously developed to be resistant to the anti-EGFR monoclonal antibody cetuximab [31], [32]), HNSCC lines SCC6 and SCC1, and the CRC lines LoVo and CaCO2 (**Figure 1A** **)**. Results from this experiment indicated that HER3 was expressed broadly across a variety of tumor types. Further, isolation of nuclei from H226^R^, SKBr3 and MCF-7 cells indicated that full-length HER3 (∼185 kDa) could be detected in the nucleus**,** whereas nuclear HER3 was undetectable in the HER3 low-expressing breast cancer cell line BT549 (**Figure 1B** **)**. The plasma membrane associated proteins clathrin and dynamin, as well as the endoplasmic reticulum (ER) associated protein calnexin, were used to demonstrate nuclear fraction (Nuc) purity from other membrane-bound proteins and ER proteins. Additionally, the cytoplasmic protein α-tubulin and the nuclear protein Histone H3 were used as non-nuclear fraction (NN) and Nuc purity controls.

**Figure 1:** The HER3 receptor is localized to the nucleus in its full-length form. **A. HER3 is expressed in numerous cancer cell lines.** Whole cell protein lysates were isolated from various breast, lung, HNSCC, and colon cancer cell lines. Lysate was fractionated on SDS-PAGE followed by immunoblotting for HER3. α-tubulin was used as a loading control. **B. HER3 is localized to the nucleus in cancer cell lines.** H226^R^, SKBr3, MCF-7, and BT549 cells were harvested for whole cell (WC), non-nuclear (NN) and nuclear (Nuc) protein, fractionated on SDS-PAGE followed by immunoblotting for HER3. Clathrin, dynamin, calnexin, α-tubulin and Histone H3 were used as loading and purity controls for the NN and Nuc fractions, respectively. **C. Specificity of nuclear HER3 by siRNA.** H226^R^ and SKBr3 cells were harvested for NN and Nuc protein 48 hr post treatment with siHER3 or non-targeting (NT) siRNA. Experimental procedure as in 1B. α-tubulin and Histone H3 were used as loading and purity controls for the NN and Nuc fractions, respectively. **D. Full-length HER3 is localized to the nucleus.** H226^R^ and SKBr3 cells were harvested for WC, NN, and Nuc lysate. WC lysates were harvested 48 hr post treatment with siHER3. 250 ug of cell lysate was immunoprecipitated with an N-TERM HER3 antibody or human IgG control. The immunoprecipitates were fractionated on SDS-PAGE followed by immunoblotting for HER3 with a C-TERM antibody.

RETRACTED

To validate the specificity of the nuclear HER3 signal detected in **Figure 1B** **,** we used siRNA to knockdown HER3 expression and subsequently performed nuclear fractionation in H226^R^ and SKBr3 cell lines. The knockdown of HER3 led to a loss of the 185 kDa band in both the NN and Nuc fractions, whereas vehicle (V) and non-targeting (NT) siRNA did not affect HER3 expression (**Figure 1C** **)**; this demonstrates that the nuclear 185 kDa band detected is specific for HER3.

To further show that nuclear HER3 is full-length within the nucleus, we performed IP analysis using an antibody that recognizes the extracellular N-terminal region of HER3 (N-TERM) followed by immunoblot analysis with an antibody that recognizes the C-terminal region of HER3 (C-TERM) in the presence of HER3 siRNA. HER3 could be effectively immunoprecipitated with an N-TERM antibody from whole cell lysate (WC) in both H226^R^ and SKBr3 cells, which was prevented upon knockdown of HER3 with siRNA **(** **Figure 1D** **)**. IP analysis was further performed from NN and Nuc lysate harvested from H226^R^ and SKBr3 cells using the same N-TERM HER3 antibody (**Figure 1D**), demonstrating that full-length HER3 can be extracted from the Nuc fraction.

Confocal immunofluorescent (IF) microscopy was used to visualize HER3 localization in H226^R^ and SKBr3 cells using both C-TERM and N-TERM HER3 antibodies (**Figure 2**). HER3 was detected using an Alexa Fluor-546 labeled secondary antibody (visualized in red). Merging DAPI and 546 labeled HER3 yielded distinct nuclear HER3 signals in both cell lines with little bleed through from the 405 laser (used to visualize DAPI). Additionally, we detect minimal HER3 staining in the HER3 low expressing cell line BT549, demonstrating specificity for the HER3 primary antibodies. These data demonstrate that full-length HER3 is localized to the nucleus in various cancer cell lines.

**Figure 2:** Confocal Immunofluorescent staining of nuclear HER3. C-TERM and N-TERM HER3 antibodies were used to visualize HER3 localization in H226^R^, SKBr3, and BT549 cells. Alexa Fluor-546 secondary antibody was used to visualize HER3 (RED) and DAPI was used to visualize the nucleus (BLUE). Merged images were magnified to depict the nuclear localization of HER3 (see white arrows). Magnification 600X.

### The C-terminus of HER3 Contains a Strong Transactivation Domain

Recent studies have demonstrated that EGFR, HER2, and small splice variants of HER3 can function as co-transcriptional activators for various gene targets [4], [5], [8], [30]. The weak tyrosine kinase activity of HER3 and its role in resistance to numerous therapeutic agents promoted our investigation into the non-kinase functions of HER3, including its transactivation potential. To investigate this, we utilized the Gal4/luciferase assay system, where the Gal4 DNA binding domain (Gal4DBD) of the yeast transcription factor Gal4 was fused to the intracellular domain (ICD), juxtamembrane and tyrosine kinase domain (JKD), and the C-terminal domain (CTD) of HER3. As a control for this assay, the EGFR-ICD and CTD were fused to the Gal4DBD as performed by Lin et al [6] (**Figure 3A**). While the EGFR-CTD strongly activated Gal4 UAS-luciferase, the EGFR-ICD was less capable of transactivating UAS-luciferase (**Figure 3B**) recapitulating previous findings [6]. The overexpression of the HER3-CTD led to strong transactivation of Gal4 UAS-luciferase (∼8.7 fold) in CHOK1 cells, while the HER3-ICD and HER3-JKD constructs resulted in minimal luciferase activity that were not statistically different from luciferase detected from the Gal4DBD vector control (**Figure 3C**). To broaden the scope of this finding we transfected two other cell lines and observed similar results (**Figure 3D**). Overall, these data demonstrate that the HER3-CTD contains strong transactivation potential.

RETRACTED

**Figure 3:** The C-terminus of HER3 contains a strong transactivation domain. **A. EGFR intracellular domain (ICD) map and plasmid validation.** The intracellular domain (ICD) and C-terminal domain (CTD) of EGFR were fused to the Gal4 DNA binding domain (Gal4DBD). CHOK1 cells were transfected with each construct for 48 hr prior to harvesting WC lysate and fractionation on SDS-PAGE followed by immunoblotting for EGFR and Gal4DBD. EGFRWT vector was transfected into CHOK1 cells as a positive control. α-tubulin was used as a loading control**. B. EGFR-CTD contains strong transactivation potential.** CHOK1 cells were transfected with EGFR-ICD or EGFR-CTD constructs, UAS-luciferase and Tk-*Renilla* reporter plasmids for 48 hr prior to quantification by dual luciferase assay (n = 3). The graphs are representative of four independent experiments. **C. HER3-ICD map and plasmid validation.** The HER3- ICD, juxtamembrane and tyrosine kinase domain (JKD), and CTD were fused to the Gal4DBD. Transfection was performed the same as in 1A and immunoblot analysis was performed for HER3 and Gal4DBD. HER3WT was transfected into CHOK1 cells as a positive control. α-tubulin was used as a loading control. **D. HER3-CTD contains strong transactivation potential.** CHOK1, H226^R^, and SKBr3 cells were transfected with HER3-ICD, HER3-JKD, and HER3-CTD constructs, UAS-luciferase and Tk-*Renilla* reporter plasmids for 48 hr prior to quantification by dual luciferase assay (n = 3). The graphs are representative of four independent experiments. Luciferase activity was normalized to DNA content, protein content, and the expression of *Renilla* luciferase in all assays. Luciferase activity detected for each construct was normalized to the Gal4DBD vector control. Data points are represented as mean+/−s.e.m. p<0.05. TM (transmembrane); JM (juxtamembrane); KD (kinase domain).

RETRACTED

### Minimal Mapping of the HER3 C-terminus Demonstrates the Existence of a Bipartite Transactivation Domain

To further understand the capability of HER3 to function as a transcription factor, we sought to map the minimal C-terminal TADs. Previous reports suggest that TADs often contain proline-rich regions [42], [43]; therefore, we analyzed the CTD of HER3 for proline-rich sequences. Two C-terminal proline-rich regions were identified, one between amino acids 1,142–1,150, and a second between amino acids 1,208–1,214. To investigate if these proline-rich sequences function as TADs both regions were deleted from the HER3-CTD (**Figure 4A**). The ability for HER3-CTD deleted of proline-rich region 1 (CTDΔP_1_), proline-rich region 2 (CTDΔP_2_), or both proline-rich regions (CTDΔP_1_ΔP_2_) to transactivate Gal4 UAS-luciferase was not statistically different from that of the HER3-CTD (**Figure 4B** **)**. These data suggest that HER3’s C-terminal proline-rich regions do not confer strong transactivation potential and therefore may not function as prominent TADs.

**Figure 4:** Minimal mapping of the HER3 C-terminus demonstrates the existence of a bipartite transactivation domain. **A. HER3-CTD proline deletion mapping and validation.** The HER3-CTD deleted of proline-rich region 1 (CTDΔP_1_), proline-rich region 2 (CTDΔP_2_), and both regions (CTDΔP_1_ΔP_2_) were fused to the Gal4DBD. CHOK1 cells were transfected with each construct for 48 hr prior to harvesting WC lysate and fractionation on SDS-PAGE followed by immunoblotting for Gal4DBD. **B. The HER3-CTD proline-rich regions do not function as prominent TADs.** CHOK1 cells were transfected with the HER3-CTD, CTDΔP_1_, CTDΔP_2_, or CTDΔP_1_ΔP_2_, UAS-luciferase and Tk-*Renilla* reporter plasmids for 48 hr prior to quantification by dual luciferase assay (n = 6). The graph is representative of three independent experiments. **C. HER3-CTD minimal transactivation domain mapping and validation.** Nine consecutive regions of the HER3-CTD of increasing length were fused to the Gal4DBD (CTD_1_-CTD_9_). CHOK1 cells were transfected with each construct for 48 hr prior to harvesting WC lysate and fractionation on SDS-PAGE followed by immunoblotting for Gal4DBD. **D. HER3-CTD contains two regions with strong transactivation potential.** CHOK1 cells were transfected with CTD_1_-CTD_9_, UAS-luciferase and Tk-*Renilla* reporter plasmids for 48 hr prior to quantification by dual luciferase assay (n = 3). The graph is representative of three independent experiments. **E. HER3-CTD bipartite deletion mapping and validation.** The regions with strong transactivation potential were deleted from the HER3-CTD, denoted as CTDΔB_1_ and CTDΔB_2_. The double deletion mutant CTDΔB_1_ΔB_2_ was also constructed. As a control, a region of similar size to B_1_ and B_2_ was deleted, denoted as CTDΔR_1_. CHOK1 cells were transfected with each construct for 48 hr prior to harvesting WC lysate and fractionation on SDS-PAGE followed by immunoblotting for Gal4DBD. **F. HER3 contains a strong bipartite C-terminal TAD.** CHOK1 cells were transfected with CTDΔB_1_, CTDΔB_2_, CTDΔB_1_ΔB_2_, or CTDΔR_1_, UAS-luciferase and Tk-*Renilla* reporter plasmids for 48 hr prior to quantification by dual luciferase assay (n = 6). The graph is representative of four independent experiments. Luciferase activity was normalized to DNA content, protein content, and the expression of *Renilla* luciferase in all assays. Luciferase activity detected for each construct was normalized to the pM Gal4DBD vector control. Data points are represented as mean +/− s.e.m. P<0.05.

RETRACTED

To identify HER3 TADs we next constructed a series of nine Gal4DBD HER3-CTD mapping mutants, where small regions of the HER3-CTD were sequentially added back to each construct until the entire HER3-CTD was restored (**Figure 4C**). The transactivation capability of each mapping mutant (CTD_1_–CTD_9_) was then tested via Gal4 UAS-luciferase assays in CHOK1 cells (**Figure 4D**). The CTD_1_ and CTD_2_ constructs had minimal transactivation activity (similar activity to the Gal4DBD vector control), while CTD_3–5_ expression yielded slightly more transactivation activity. However, CTD_6_ demonstrated a 5.0 fold increase in Gal4 UAS-luciferase activation (∼3.0 fold higher than CTD_5_, p<0.001). The CTD_7_ construct demonstrated similar transactivation activity to CTD_6_, while CTD_8_ displayed a 7.5 fold increase in Gal4 UAS-luciferase activation (∼2.5 fold higher than CTD_7_, p<0.01), which recapitulated the luciferase activity detected from the full-length HER3-CTD. The CTD_9_ construct exhibited similar transactivation activity to CTD_8_ and the full-length HER3-CTD. These data suggest that the HER3-CTD contains two prominent TADs, one between CTD_5_ and CTD_6_, and a second between CTD_7_ and CTD_8_.

RETRACTED

To validate the bipartite TAD identified in **Figure 4D**, both regions were deleted from the HER3-CTD (**Figure 4E**). The first deletion mutant consisted of the region located between CTD_5_ and CTD_6_ (amino acids 1,215–1,248) denoted as CTDΔB_1_ and the second deletion mutant consisted of the region located between CTD_7_ and CTD_8_ (amino acids 1,281–1,302) denoted as CTDΔB_2_. The double bipartite deletion mutant was also constructed, denoted as CTDΔB_1_ΔB_2_. To ensure that the B_1_ and B_2_ regions are specific TADs, we also deleted one region in the HER3-CTD of approximately the same size as B_1_ and B_2_ denoted as CTDΔR_1_ (**Figure 4E**). While the HER3-CTD transactivated Gal4 UAS-luciferase 7.4 fold higher than the Gal4DBD vector control, CTDΔB_1_ and CTDΔB_2_ led to statistically significant reductions in UAS-luciferase activity (3.2 and 2.0 fold decreases), while the CTDΔB_1_ΔB_2_ demonstrated the greatest reduction (4.9 fold decrease) (**Figure 4F**). The CTDΔR_1_ was not hindered in its ability to transactivate UAS-luciferase, demonstrating specificity of the B_1_ and B_2_ regions. Collectively, these data demonstrate that the B_1_ and B_2_ regions contain the majority of HER3’s transactivation potential.

### Nuclear HER3 can Associate with a 122 bp Region of the Cyclin D1 Promoter

To understand how the identified bipartite TAD influences nuclear HER3’s transcriptional functions we sought to identify a nuclear HER3 gene target. Since full-length nuclear EGFR and HER2 and a nuclear variant of HER3 have been shown to associate with the cyclin D1 promoter [6]–[8], we hypothesized that full-length nuclear HER3 would be similarly associated. As a control, we first validated via chromatin immunoprecipitation (ChIP) analysis that EGFR and HER2 can associate with a 122 bp region of the cyclin D1 promoter (-33 - +89) approximately 6.8 fold (EGFR) and 9.4 fold (HER2) higher than an IgG control **(** **Figure 5A** **)**. Additionally, DNA affinity precipitation assays (DAPA) were performed using a biotinylated 122 bp cyclin D1 promoter probe. Both EGFR and HER2 associated with the cyclin D1 promoter probe while lysate incubated with beads only lacked association.

**Figure 5:** HER3 can associate with the cyclin D1 promoter. **A. Nuclear EGFR and HER2 associate with the cyclin D1 promoter.** ChIP using an anti-EGFR, anti-HER2, or normal rabbit IgG antibody was performed with SKBr3 cells and isolated DNA was subsequently used for qPCR with primers flanking the 122 bp cyclin D1 promoter region (n = 3). qPCR specificity for the 122 bp cyclin D1 promoter was confirmed by agarose gel electrophoresis of semi-qPCR products. DAPA analysis was performed using a biotinylated 122 bp cyclin D1 promoter probe incubated with 400 ug of nuclear lysate harvested from SKBr3 cells. Bound proteins were isolated with streptavidin agarose beads and subsequently fractionated on SDS-PAGE followed by immunoblotting for EGFR or HER2. Nuclear lysate incubated with beads only lacked association. **B. Nuclear HER3 can associate with the cyclin D1 promoter.** ChIP using a N-TERM anti-HER3 or a human IgG antibody was performed with H226^R^, SKBr3, and BT549 cells. qPCR was performed as in 5A. **C. HER3 can associate with a cyclin D1 promoter probe.** DAPA analysis was performed using nuclear lysate harvested from H226^R^, SKBr3, MCF-7, and BT549 cells as in 5A. Proteins isolated from the probe were subsequently fractionated on SDS-PAGE followed by immunoblotting for HER3. **D. HER3 association with the cyclin D1 promoter probe is specific.** DAPA analysis was performed as in 5A using nuclear lysate harvested from H226^R^, SKBr3, MCF-7, and BT549 cells transfected with either non-targeting (NT) or HER3 siRNA for 48 hr. Proteins isolated from the probe were subsequently fractionated on SDS-PAGE followed by immunoblotting for HER3. All data points for ChIP are represented as mean +/− s.e.m and normalized to the IgG control. P<0.05.

RETRACTED

Next, ChIP was performed using an N-TERM HER3 antibody in H226^R^, SKBr3, and BT549 cells. Full-length HER3 associated with the 122 bp region of the cyclin D1 promoter in both H226^R^ (3.2 fold) and SKBr3 (5.6 fold) cells while HER3 association with cyclin D1 could not be detected in the HER3 low expressing cell line BT549 (**Figure 5B**). Additionally, HER3 associated with the cyclin D1 promoter probe in a DAPA assay (**Figure 5C** **)**. Detection of HER3 in this assay was specific because siHER3 knockdown studies demonstrated loss of probe binding (**Figure 5D**). Collectively, these data demonstrate that nuclear HER3 can associate with a 122 bp region of the cyclin D1 promoter.

### Nuclear HER3 can Regulate the Transcription of a 122 bp Region of the Cyclin D1 Promoter via its Bipartite Transactivation Domain

Since full-length nuclear HER3 can associate with a 122 bp region of the cyclin D1 promoter, we sought to understand its ability to regulate this region. To do this, the 122 bp region of the cyclin D1 promoter was cloned into a luciferase reporter construct. In **Figure 6A** **,** the knockdown of HER3 expression using siRNA decreased cyclin D1-promoter luciferase 24% in H226^R^, 35% in SKBr3, and 27% in MCF-7 cells compared to cells transfected with NT siRNA. Lysate from the luciferase assay was used to confirm the knockdown of HER3 expression. In **Figure 6B** **,** HER3 was overexpressed in SCC6, HCC1954, SKBr3, and BT474 cells, where cyclin D1 promoter-luciferase activity was significantly increased (90%, 50%, 35%, and 65% respectively). Nuclear lysate was obtained to validate the presence of nuclear HER3 upon overexpression. Overall, these experiments demonstrate that HER3 can influence the activation of a 122 bp region of the cyclin D1 promoter in numerous cell lines.

RETRACTED

**Figure 6:** Nuclear HER3 can regulate a minimal region of the cyclin D1 promoter via its bipartite transactivation domain. **A. HER3 knockdown decreases the activation of the cyclin D1 promoter.** H226^R^, SKBr3, and MCF-7 cells were incubated with non-targeting (NT) or HER3 siRNA for 24 hr followed by transfection with the 122 bp cyclin D1 promoter-luciferase and Tk-*Renilla* reporter plasmids for 48 hr prior to quantification by dual luciferase assay (n = 6). Percent decreases in cyclin D1 promoter-luciferase activity were normalized to NT transfected cells. The graph is representative of three independent experiments. Luciferase lysate was fractionated on SDS-PAGE followed by immunoblotting for HER3. **B. HER3 overexpression activates the cyclin D1 promoter.** SCC6, HCC1954, SKBr3, and BT474 cells were transfected with HER3WT or control vector, 122 bp cyclin-D1-luciferase and Tk-*Renilla* reporter plasmids for 48 hr prior to quantification by dual luciferase assay (n≥3). Percent increases in cyclin D1-promoter luciferase were normalized to vector transfected cells. The graph is representative of three independent experiments. Nuclear lysate was harvested from each cell line and fractionated on SDS-PAGE followed by immunoblotting for HER3. α-tubulin and Histone H3 were used as loading and purity controls for the Nuc fraction. **C. HER3ΔB_1_ΔB_2_ overexpression can prevent the activation of the cyclin D1 promoter while HER3DM remains functional.** SCC6, BT474 and HCC1954 cells were transfected with HER3WT, HER3DM, HER3ΔB_1_ΔB_2_ or control vector, the 122 bp cyclin-D1-luciferase and Tk-*Renilla* reporter plasmids for 48 hr prior to quantification by dual luciferase assay (n≥3). Percent increases in cyclin D1 promoter-luciferase were normalized to vector transfected cells. The graph is representative of seven independent experiments. **Inset 1:** CHOK1 cells were transfected with HER3WT, HER3ΔB_1_ΔB_2_ or control vector for 48 hr prior to harvesting NN and Nuc protein, fractionation on SDS-PAGE followed by immunoblotting for HER3. α-tubulin and Histone H3 were used as loading and purity controls for Nuc fraction. **Inset 2:** CHOK1 cells were transfected with HER3WT, HER3DM, HER3ΔB_1_ΔB_2_ or control vector and stimulated for 40 min with 5 nM neuregulin-1. Whole cell lysate was fractionated on SDS-PAGE followed by immunoblotting for indicated proteins. **D. HER3 knockdown decreases cyclin D1 expression.** SCC6 and BT474 cells were incubated with NT or HER3 siRNA for 48 hr prior to harvesting RNA. The mRNA expression of cyclin D1 was determined by qPCR (n = 3) and normalized to NT transfected cells. The graph is representative of two independent experiments. **E. The overexpression of HER3WT enhances cyclin D1 expression while HER3ΔB_1_ΔB_2_ is hindered.** SCC6 and BT474 cells were transfected with HER3WT, HER3ΔB_1_ΔB_2_ or control vector for 72 hr prior to harvesting RNA. The mRNA expression of cyclin D1 was determined by qPCR (n = 3) and normalized to vector transfected cells. The graph is representative of four independent experiments. All luciferase values were normalized to DNA content, protein content, and the expression of *Renilla* luciferase. All data points are represented as mean +/− s.e.m. P<0.05.

RETRACTED

Next, we measured the ability for full-length HER3 deleted of both the B_1_ and B_2_ regions (denoted as HER3ΔB_1_ΔB_2_) to transactivate cyclin D1 promoter-luciferase. While the overexpression of wild-type HER3 (HER3WT) led to increases in cyclin D1 promoter-luciferase activity in SCC6, BT474 and HCC1954 cells (97%, 63% and 30% respectively), the overexpression of HER3ΔB_1_ΔB_2_ was hindered in its ability to transactivate cyclin D1 in all cell lines (10%, 14% and 0% respectively) (**Figure 6C**). Analysis of the B_1_ and B_2_ regions yielded the presence of two tyrosine residues: tyrosine 1222 located in B_1_, and tyrosine 1289 located in B_2_. To verify that the loss of luciferase activity by HER3ΔB_1_ΔB_2_ was not due to altered signaling dependent on these tyrosines, we tested the ability for a double tyrosine mutant (HER3 Y1222F/Y1289F denoted as HER3DM) to transactivate cyclin D1 promoter-luciferase (**Figure 6C**). The overexpression of HER3DM in all cell lines demonstrated a minor reduction in functionality as compared to HER3WT in this assay (85%, 55%, and 27% respectively); however, the luciferase values between HER3WT and HER3DM were not statistically different from one another in each cell line (**Figure 6C**). Additionally, both HER3WT and HER3ΔB_1_ΔB_2_ were effectively nuclear localized (**Inset 1,** **Figure 6C**) and the activation of the downstream signaling molecule AKT was not affected in all mutants (**Inset 2,** **Figure 6C**). These data suggest that the alterations in cyclin D1 luciferase observed upon overexpression of HER3ΔB_1_ΔB_2_ were not due to a loss of nuclear HER3 localization or changes in AKT activity.

To further understand if the B_1_ and B_2_ TADs are required for HER3 induced cyclin D1 expression, we performed quantitative PCR (qPCR) to measure cyclin D1 transcripts after treatment with siHER3 (**Figure 6D**) or overexpression of HER3WT and HER3ΔB_1_ΔB_2_ (**Figure 6E**). siRNA knockdown of HER3 in H226^R^ and MCF-7 cells led to significant decreases in cyclin D1 expression (39% and 50% downregulation respectively) as compared to NT treated cells (**Figure 6D**). Importantly, the overexpression of HER3WT vs. HER3ΔB_1_ΔB_2_ in SCC6 and BT474 cells demonstrated that HER3WT could significantly enhance cyclin D1 expression (92% and 35% upregulation respectively), while the HER3ΔB_1_ΔB_2_ mutant was severely hindered at doing so (8% and 1% upregulation respectively) (**Figure 6E**). The minor increases in cyclin D1 transcripts detected upon HER3ΔB_1_ΔB_2_ overexpression were not statistically different from vector transfected cells. Collectively, these data suggest that nuclear HER3 can regulate cyclin D1 expression, in part, through its B_1_ and B_2_ TADs.

RETRACTED

### An Intracellular Domain Mutant of HER3 can Regulate the Transcription of Cyclin D1 via its Bipartite Transactivation Domain

To further ensure that nuclear HER3, rather than classical signaling emanating from membrane-bound HER3, functions in the regulation of cyclin D1 we created intracellular domain (ICD) truncation mutants of HER3 that lack both the N-terminus and the transmembrane domain (**Inset 1,** **Figure 7A** **for illustration**). HER3WT-ICD (denoted as WT-ICD) and HER3ΔB_1_ΔB_2_-ICD (denoted as ΔB_1_ΔB_2_-ICD) were overexpressed in SCC6, BT474, and HCC1954 cells alongside the 122 bp cyclin D1 promoter-luciferase construct. While the overexpression of WT-ICD led to increases in cyclin D1 promoter-luciferase activity (60%, 25% and 94% respectively), the overexpression of ΔB_1_ΔB_2_-ICD was hindered in its ability to transactivate cyclin D1 in all cell lines (12%, 8% and 11% respectively) (**Figure 7A**). Additionally, both WT-ICD and ΔB_1_ΔB_2_-ICD were effectively nuclear localized (**Inset 2,** **Figure 7A**). Next, qPCR was performed to assess the ability for each ICD mutant to augment cyclin D1 expression (**Figure 7B**). The overexpression of WT-ICD in SCC6 and BT474 cells significantly enhanced cyclin D1 expression (200% and 40% upregulation respectively), while ΔB_1_ΔB_2_–ICD was hindered at doing so (5% and 12% upregulation respectively). The minor increases in cyclin D1 promoter-luciferase and transcripts detected upon HER3ΔB_1_ΔB_2_ overexpression were not statistically different from vector transfected cells. Collectively, these data indicate that HER3 depleted of its membrane-bound functions can effectively regulate the cyclin D1 promoter through its bipartite TAD.

RETRACTED

**Figure 7:** An intracellular domain (ICD) mutant of HER3 can regulate a minimal region of the cyclin D1 promoter via its bipartite transactivation domain. **A. HER3WT ICD (WT-ICD) can activate the cyclin D1 promoter while HER3ΔB_1_ΔB_2_-ICD (ΔB_1_ΔB_2_-ICD) is hindered.** SCC6, BT474, and HCC1954 cells were transfected with WT-ICD, ΔB_1_ΔB_2_-ICD or control vector, the 122 bp cyclin D1-luciferase and Tk-*Renilla* reporter plasmids for 48 hr prior to quantification by dual luciferase assay (n≥3). Percent increases in cyclin D1 promoter-luciferase were normalized to vector transfected cells. The graph is representative of three independent experiments. **Inset 1:** Illustration of both the WT-ICD and ΔB_1_ΔB_2_-ICD constructs. **Inset 2:** CHOK1 cells were transfected with WT-ICD and ΔB_1_ΔB_2_-ICD for 48 hr prior to harvesting NN and Nuc protein, fractionation on SDS-PAGE followed by immunoblotting for HER3. α-tubulin and Histone H3 were used as loading and purity controls for Nuc fraction. **B. The overexpression of WT-ICD can enhance cyclin D1 expression while ΔB_1_ΔB_2_-ICD is hindered.** SCC6 and BT474 cells were transfected with WT-ICD, ΔB_1_ΔB_2_-ICD or control vector for 48 hr prior to harvesting RNA. The mRNA expression of cyclin D1 was determined by qPCR (n = 3) and normalized to vector transfected cells. The graph is representative of three independent experiments. All luciferase values were normalized to DNA content, protein content, and the expression of *Renilla* luciferase. All data points are represented as mean +/− s.e.m. P<0.05. ICD (intracellular domain).

## Discussion

To date, all HER family RTKs have been shown to be nuclear localized in primary tumor tissues and cancer cell lines where they can function as co-transcription factors [4], [5]. The nuclear expression of both EGFR and HER3 have been correlated with worse disease prognosis in specific cancers [9]–[11], [13], [29], and nuclear EGFR has been shown to enhance resistance to various therapeutic agents [4], [5]. These findings highlight the need to better understand nuclear HER family function. In the current study, we sought to identify the regions on the HER3 receptor that function as TADs to enhance the understanding of HER3’s transcriptional functions. To identify HER3 C-terminal TADs, various regions of the HER3 CTD were fused to the Gal4DBD and tested for their ability transactivate Gal4 UAS-luciferase. Two regions of prominent transactivation potential were identified (B_1_ and B_2_) via this method and were further shown to impact nuclear HER3’s ability to regulate both the cyclin D1 promoter and mRNA expression.

To date, several investigators have identified full-length nuclear EGFR and HER2 in different tumor types [5], [44]. In the current report, we detected nuclear HER3 in its full-length form with both N- and C- terminal HER3 antibodies (**Figure 1** **and** **2** **)**. Additionally ChIP analysis was performed using an N-terminal HER3 antibody (**Figure 5**). In 2002, Offterdinger et al. observed full-length nuclear HER3 in human breast cancer MTSV1-7 cells [28], which was validated by Koumakpayi et al. in multiple prostate cancer cell lines [29]. Additionally, using both fluorescently labeled HER3 and cell fractionation techniques, Tao et al. demonstrated that full-length HER3 homodimers were highly localized to the nucleus in various cell models [45]. Recently, alternative splice variants of HER3 have been discovered to be nuclear localized, including an 80-kDa fragment in H358 lung cancer cells [8], and a 50-kDa fragment in rat Schwann cells [30]. In the present study, an 80-kDa fragment of HER3 was detected in whole cell lysate from some cell lines, while a 50-kDa fragment was undetectable (data not shown). Thus, in the current study the predominant form of nuclear HER3 detected was that of the full-length receptor.

RETRACTED

In 2001, a pioneering study by Lin et al. demonstrated that the C-terminus of EGFR (EGFR-CTD) contained strong transactivation potential through the use of a Gal4 UAS-chloramphenicol transferase reporter assay [6], while the EGFR-ICD and EGFR-JKD constructs elicited minimal activation. In the current study we identified that the HER3-CTD also contained strong transactivation potential, similar to that of the EGFR-CTD, while the HER3-ICD and HER3–JKD constructs had minimal activity (**Figure 3**). Lin et al. hypothesized that the EGFR-JKD may contain negative regulatory sites that hinder the EGFR-CTD from functioning as a transcriptional co-activator [6]. The HER3-JKD may also contain negative regulatory sites, and therefore may inhibit the HER3-CTD from functioning in a Gal4 UAS-luciferase assay. Further experimentation is needed to identify these putative negative regulatory sites and their influence on HER3-CTD function.

TADs of transcription factors often contain proline and acidic amino acid rich regions that help recruit proteins necessary for transcription [38], [43]. To define HER3’s TADs, we first identified two prominent C-terminal proline-rich sequences (**Figure 4A**). When the proline-rich sequences were deleted from the HER3-CTD a significant change in Gal4 UAS-luciferase activity was not observed, suggesting that these regions do not function as prominent TADs (**Figure 4B**). Through sequential mapping studies we found two independent regions (B_1_ and B_2_) on the HER3-CTD that most prominently activated Gal4 UAS-luciferase (**Figure 4C–4F**). These regions demonstrated specificity because deletion of another region (R_1_) of similar size did not affect Gal4 UAS-luciferase activity (**Figure 4F**). Motif analysis of this bipartite region did not yield the presence of any known TAD sequence, however various transcription factors contain bipartite TADs, examples including p53 and CREB [46], [47]. Research over the last two decades has demonstrated that TADs are not necessarily rich in any particular sequence, and that TADs have high diversity of sequence and domain structure, unlike the uniform sequence and structure of DBDs [43], [48], [49]. While the bipartite region discovered accounted for ∼66% of HER3’s transactivation potential in a Gal4 UAS-luciferase assay, it did not recapitulate the full activity detected from the entire HER3-CTD, and therefore other CTD regions may function as less prominent TADs.

RETRACTED

To identify how B_1_ and B_2_ influence nuclear HER3 function, we first demonstrated that HER3 can bind to a 122 bp region of the cyclin D1 promoter, a region that was originally found to associate with nuclear EGFR [6]. Interestingly, EGFR, HER2, and HER3 all associated with this relatively small promoter region in SKBr3 cells (**Figure 5**). Whether HER family dimers exist in the nucleus and function together as co-transcription factors has yet to be determined. We further demonstrate that HER3 lacking the B_1_ and B_2_ regions (HER3ΔB_1_B_2_) had either reduced ability or an inability to transactivate cyclin D1 promoter-luciferase and cyclin D1 expression in multiple cell lines (**Figure 6**), suggesting that these regions function as prominent TADs. SCC6 and BT474 cells express endogenous HER3 (See **Figure 1A**) and therefore the slight increases in reporter activity detected upon overexpression of HER3ΔB_1_ΔB_2_ may have been due to activation by endogenous nuclear HER3. Additionally, both HER3WT and HER3ΔB_1_ΔB_2_ were effectively localized to the nucleus (**Inset 1,** **Figure 6C**). Therefore, the lack of cyclin D1 promoter-luciferase detected upon HER3ΔB_1_ΔB_2_ overexpression was likely due to its inability to function in the nucleus rather than impairment in nuclear translocation. The specific transcription factors that associate with nuclear HER3 is under current investigation, but we speculate that HER3ΔB_1_ΔB_2_ is deficient in the proper association and/or recruitment of these factors. Collectively, these data suggest that the B_1_ and B_2_ regions of HER3 function as TADs.

One of the major hurdles in the study of nuclear RTKs is to experimentally isolate their nuclear functions from plasma membrane-bound functions. To ensure that the loss of cyclin D1 promoter- luciferase activity detected upon overexpression of HER3ΔB_1_ΔB_2_ was due to deficiency in nuclear HER3 functions the tyrosine residues located in the B_1_ and B_2_ regions known to play a role in activating signaling cascades were mutated. HER3 mutated at both tyrosine 1222 and 1289 (HER3DM) was only slightly hindered in the activation of the cyclin D1 promoter, unlike HER3ΔB_1_ΔB_2_, and both HER3DM and HER3ΔB_1_ΔB_2_ were still capable of activating HER3’s downstream effector kinase AKT (**Inset 2,** **Figure 6C**). To further validate that the regulation of cyclin D1 was not a result of classical membrane-bound functions of HER3, ICD mutants of HER3 were created in which HER3WT and HER3ΔB_1_ΔB_2_ were deleted of both the N-terminus and transmembrane domain (**Figure 7**). The WT-ICD, which cannot be localized at the plasma membrane or serve as a dimerization partner to activate classical signaling pathways, was still capable of regulating cyclin D1 luciferase activity and mRNA expression. This finding falls in line with the identified HER3 C-terminal splice variants that have been shown to function as co-transcription factors [8], [30]. Importantly, ΔB_1_ΔB_2_-ICD was hindered in cyclin D1 regulation, further supporting the role of these TADs in influencing nuclear HER3 transcriptional function. We speculate that the minor increases in luciferase and mRNA expression observed upon ΔB_1_ΔB_2_-ICD overexpression may emanate from endogenous HER3 in SCC6 and BT474 cells and/or the residual transcriptional activity remaining on the C-terminus of the ΔB_1_ΔB_2_-ICD. Collectively, these data suggest that the loss of cyclin D1 promoter-luciferase activity and mRNA expression was not due to modulation of signaling pathways emanating from membrane-bound HER3, but likely due to an inability for HER3ΔB_1_ΔB_2_ to function as a co-transcription factor.

RETRACTED

To date, various functions of nuclear localized HER family receptors have been identified. The present study is the first to map specific TADs on a nuclear HER family member, and further TAD mapping studies of both HER2 and EGFR are underway. These studies are important because it is becoming increasingly apparent that nuclear HER family transcriptional functions play a role in cancer biology and that these functions may be independent of their kinase activity [4], [5]. The current study supports these findings because 1) HER3 lacks high levels of kinase activity, and 2) nuclear HER3 regulation of cyclin D1 was independent of plasma membrane-bound HER3 functions and AKT signaling. Since the kinase functions of HER family members may not be solely responsible for the tumorigenic properties of these receptors, the identification of HER family TADs may serve as a map to better target nuclear HER functions in the future.
